The article "SOX2 Enhances the Migration and Invasion of Ovarian Cancer Cells via Src Kinase" was retracted in 2023. Reasons: errors in the images; duplicated images; overlap with earlier publications; original data or images not available.

# SOX2 Enhances the Migration and Invasion of Ovarian Cancer Cells via Src Kinase

**DOI:** 10.1371/journal.pone.0099594

**Published:** 2014-06-17

**Authors:** Xiaojie Wang, Xiaoning Ji, Jiazhou Chen, Dong Yan, Zhenbo Zhang, Qifeng Wang, Xiaowei Xi, Youji Feng

**Affiliations:** 1 Department of Obstetrics and Gynecology, Shanghai Jiao Tong University Affiliated First People's Hospital, Shanghai, China; 2 Department of Pathology, Fudan University Shanghai Cancer Center, Shanghai Medical College, Fudan University, Shanghai, China; Thomas Jefferson University, United States of America

## Abstract

Ovarian cancer is the leading cause of death among gynecologic cancers and is the fifth leading cause of all cancer-related deaths among women. The development of novel molecular targets is therefore important to many patients. Recently, the SRY-related transcription factor SOX2 has been widely reported to be involved in multiple pathophysiological diseases, including maintenance of stem cell characteristics and carcinogenesis. Up to now, SOX2 has been mainly shown to promote the development of cancer, although its inhibitory roles in cancer have also been reported. However, the role of SOX2 in ovarian cancer is largely unknown. In the present study, we detected the expression of SOX2 in 64 human serous ovarian carcinoma (SOC) tissues and paired corresponding metastatic specimens using immunohistochemistry. The results showed that the expression of SOX2 in primary tumors is much lower than that in the corresponding metastatic lesions. We further found that SOX2 overexpression promotes proliferation, migration and invasion, while inhibiting adhesion abilities of SOC cells. Finally, we found that SOX2 targets Src kinase, a non-receptor tyrosine kinase that regulates cell migration, invasion and adhesion in SOC cells. Together, these results suggested that Src kinase is a key molecule in SOX2-mediated migration and invasion of SOC cells.

## Introduction

Ovarian epithelial cancer accounts for 80–90% of all ovarian cancers and is the leading killer among all gynecological malignancies [1]. Because of the lack of early symptoms, ovarian carcinoma is usually diagnosed at an advanced metastatic stage. Widespread metastases are the main causes for poor prognosis of patients with ovarian cancer. Although survival has increased slightly over the past 25 years, five-year survival rates remain below 50% [1]. Therefore, studying of the metastatic mechanisms of ovarian cancer has been a focus worldwide.

SOX2, a member of the SRY-related high mobility group box family, was initially found to maintain the embryonic stem cell pluripotency [2]. More recently, SOX2 was shown to be involved in a series of malignancies. Numerous studies have shown that SOX2 promotes cell proliferation, migration, invasion and tumor metastasis in several tumor types such as glioblastomas [3], colorectal cancer [4], prostate cancer [5], breast cancer [6], [7] and osteosarcomas [8]. Moreover, high expression levels of SOX2 correlate with tumor progression or poor prognosis of multiple cancers. In contrast, the tumor-suppressive role of SOX2 was also reported in gastric cancer [9], and squamous cell lung cancer [10].

The article "SOX2 Enhances the Migration and Invasion of Ovarian Cancer Cells via Src Kinase" was retracted in 2023. Reasons: errors in the images; duplicated images; overlap with earlier publications; original data or images not available.

Recently, several studies have found that SOX2 expression is significantly increased in ovarian cancer tissues compared with normal ovary tissues using immunohistochemistry [11], [12]. Multivariate analysis further demonstrated that the SOX2 overexpression is a poor prognostic factor in ovarian cancer [13], [14]. These findings suggested that SOX2 might act as a tumor-promoting gene in ovarian cancer. However, the functional roles and precise mechanisms are still elusive in ovarian cancer. To clarify the role and underlying mechanisms of SOX2 in ovarian epithelial cancer, we examined the expression of SOX2 in serous ovarian carcinoma(SOC)and matched metastatic tissues, as well as in SOC cell lines. Moreover, we analyzed the effect of the SOX2 gene on the proliferation, migration and adhesion abilities of SOC cells.

## Materials and Methods

### Human SOC samples and clinical information

SOC primary and matched metastatic tissues (omentum) were obtained from the Department of Pathology at the First People's Hospital of Shanghai. Use of the specimens was approved by the Human Investigation Ethical Committee of the First People's Hospital of Affiliated Shanghai Jiao Tong University. All these samples were obtained with written informed consent. The specific samples used in this study have been described in previous publication [15]. In total 64 serous cystadenocarcinoma with omentum metastasis (stage III) were studied. The age of patients with ovarian cancer ranged from 34 to 81 years (median of 61.2). There are 55 cases with menopause. The formaldehyde-fixed and paraffin-embedded tissue specimens from 64 cases of SOC were collected between January 2003 and December 2010. Patients with prior radiation or chemotherapy were excluded. Pathological diagnoses of the above ovarian lesions were made by two gynecological pathologists using the World Health Organization classification.

### Immunohistochemical (IHC) staining and evaluation

IHC analysis for SOX2 protein expression was carried out as previously described. Briefly, SOX2 expression was detected using a rabbit monoclonal anti-human SOX2 (Cell Signal Technology, Danvers, MA, USA). The sections were incubated with anti-SOX2 (1∶100 dilution) in a moisture chamber for 2h followed by a 60-min incubation with a biotinylated secondary antibody. The percentage of positively stained cells and the intensity of the staining in these slides were assessed in a blinded manner. Positive cells were indicated by the presence of brown staining in both the nucleus and cytoplasm. IHC results were evaluated under a light microscope and scored as follows: 0 <5% positive cells; 1 5–25% positive cells; 2 26–75% positive cells; and 3 >76% positive cells. Stain intensity was scored as: 0, no staining; 1, faint-yellow; 2, brown–yellow; and 3, dark-brown. The expression level (plus of the two scores) was classified as: - (0), +(1–2), ++(3–4), and +++(5–6). Scores ≥3 were defined as high-level expression and scores < 3 were defined as low-level expression. Individual IHC scores for each case were used for statistical analysis. All IHC slides were reviewed independently by two investigators.

The article "SOX2 Enhances the Migration and Invasion of Ovarian Cancer Cells via Src Kinase" was retracted in 2023. Reasons: errors in the images; duplicated images; overlap with earlier publications; original data or images not available.

### Cell lines and cell culture

Ovarian cancer cell lines Hey, HO8910, and HO8910-pm were obtained from the American Type Culture Collection (Manassas, VA, USA) and cultured based on the guidelines of the repository. The cells were maintained in Dulbecco's modified Eagle's medium (DMEM)/F12 supplemented with 10% fetal bovine serum (FBS). The MCV152 and Moody cell lines were kindly provided by Dr Wenxin Zheng (Arizona University, Tucson, AZ, USA). SKOV3 cells were purchased from the Beijing Union Medical College (Beijing, China). The three SOC cell lines and HEK-293T were cultured in DMEM supplemented with 10% FBS, 100 U/ml penicillin, 100 µg/ml streptomycin, sodium pyruvate and L-glutamine at 37°C with 5% CO2.

### RNA extraction and quantitative real-time PCR

Total RNA was extracted using TRIzol reagent (Invitrogen, Carlsbad. CA. USA). Complimentary DNA (cDNA) was synthesized with the Prime-Script RT reagent Kit (TaKaRa, Japan). Fold inductions were calculated using the formula 2-(ddCt) using GAPDH as an internal control gene. Real-time PCR was performed using SYBR Premix Ex Taq (TaKaRa, Japan). The gene-specific primer pairs were as follows: SOX2 (F) 5'-CGG CAA CCA GAA AAA CAG C-3', SOX2 (R) 5'-TCT CCG TCT CCG ACA AAA GT-3'; GAPDH (F) 5'-GGT GGT CTC CTC TGA CTT CAA CA-3', GAPDH (R) 5'-GTT GCT GTA GCC AAA TTC GTT GT-3'.

### Transient transfection of SOX2 small interfering RNA (siRNA) and Src siRNA

Ho8910-pm and Skov3 cells were plated in six-well plates at a density of 4×10^5^ cells/well. After 24 h of culture, the medium was replaced by Opti-MEM (Invitrogen) in the absence of antibiotics and cultured. siRNA corresponding to the gene was designed and synthesized by Genepharma (Shanghai, China). In total 100 pmol of siRNA was transfected using 5 µL of lipofectamine RNAiMax reagent (Invitrogen). After incubation for another 48 h, the treated cells were used to investigate the effect of gene depletion using Western blot analysis or transwell and adhesion assays. The siRNA sequences against SOX2 included: (1)5'-CUGCAGUACAACUCCAUGATT-3'; (2) 5'-GGACAUGAUCAGCAUGUAUTT-3'; (3)5'-CCA UGG GUU CGG UGG UCAA TT-3'. The siRNA sequences against Src included: (1) 5'-CAG GCU GAG GAG UGG UAU UTT-3'; (2) 5'-GCC UCA ACG UGA AGC ACU ATT-3'; (3) 5'-CUC GGC UCA UUG AAG ACA ATT-3'.

The article "SOX2 Enhances the Migration and Invasion of Ovarian Cancer Cells via Src Kinase" was retracted in 2023. Reasons: errors in the images; duplicated images; overlap with earlier publications; original data or images not available.

### Plasmid construction

The SOX2 ORF sequence was amplified from the SOX2 vector, which was produced by Shanghai R&S Biotechnology Co. Ltd (Shanghai, China). The integrity of the cDNA was confirmed by sequencing. The SOX2 ORF sequence was inserted into the EcoRI-BamHI site of the pWPXL plasmid and ligated into the vector (a gift from Dr. Didier Trono). The primer sequence of SOX2 included: SOX2 (F) 5'- CGC GGA TCC ATG TAC AAC ATG ATG GAG ACG GAG C-3'; SOX2 (R) 5'-CCG GAA TTC GAT TTA TCG CGT CGA CTC ACA TG-3'.

### Lentivirus production and cell transduction

The packaging plasmid psPAX2 and the envelope plasmid pMD2.G were gifts from Dr. T. Didier Trono. pWPXL-SOX2 vector was cotransfected with psPAX2 and pMD2.G into HEK293T cells using Lipofectamine2000 (Invitrogen). Viruses were harvested 48 h after transfection and viral titers were determined. Ho8910 cells were infected with 1×10^6^ recombinant lentivirus transduction units in the presence of 6 µg/mL polybrene (Sigma, MO. USA).

### Cell- extracellular matrix (ECM) adhesion assay

The ability of the ovarian carcinoma cells to adhere to ECM components was quantified as previously described [16]. 96-well plates were coated with 1 mg/ml matrigel (BD,USA), 10 µg/ml plasma fibronectin(Millipore, Billerica, MA, USA), 10 µg/ml type I collagen (Millipore, Billerica, MA, USA), 10 µg/ml laminin(Millipore, Billerica, MA, USA), or with 100 ug/ml bovine serum albumin (BSA; Sigma,USA), and incubated overnight at 4°C. Subsequently, non-specific binding sites were blocked with 1% BSA in phosphate-buffered saline (PBS) for 4 h at 37°C or overnight at 4°C, then plates were washed by PBS twice. The cells (4.0×10^4^cells/100 µl) diluted with DMEM were added to the coated 96-well plates and incubated at 37°C for 30∼60 minitus in a CO2 incubator. Non-adherent cells were removed by washing with PBS. Attached cells were analyzed using a Cell Counting Kit-8 (CCK-8, Dojindo, Kumamoto, Japan) according to the manufacturer's instructions, and the optical density was measured at 450 nm. These experiments were performed in triplicate and repeated twice.

The article "SOX2 Enhances the Migration and Invasion of Ovarian Cancer Cells via Src Kinase" was retracted in 2023. Reasons: errors in the images; duplicated images; overlap with earlier publications; original data or images not available.

### Cell proliferation assays

Cells were seeded at a density of 2000 cells per well in 96-well plates and incubated. An aliquot of 10 µl of CCK-8 was added to the wells and incubated for 2 h. The absorbance was measured at 450 nm to calculate the numbers of viable cells in each well. Each measurement was performed in triplicate and the experiments were repeated twice.

For colony formation assays, cells were seeded in six-well plates at a density of 200 cells per well and cultured at 37°C for two weeks. At the end of the incubation, the cells were fixed with 100% methanol and stained with 0.1% (w/v) Crystal Violet. Megascopic cell colonies were counted using Image-Pro Plus 5.0 software (Media Cybernetics, Bethesda, MD, USA). Each measurement was performed in triplicate and the experiments were each conducted at least three times.

### Migration and invasion assays

Cell migration assay: 4×10^4^ cells were suspended in 200 µl serum-free DMEM medium and seeded into the upper chamber of each insert. Then, 500 µL of DMEM containing 10% FBS was added to a 24-well plate. After incubation at 37°C (Ho8910: 12–14 h; Ho8910-pm:12–14 h; Skov3: 12–14 h), the cells that migrated were fixed and stained for 30 min in a 0.1% Crystal Violet solution in PBS.

Cell invasion assay: chambers were uniformly covered with 60 µL Matrigel diluted with DMEM to a certain percentage and incubated at 37°C for 2–4 h. Then, 4×10^4^ cells were suspended in 200 µL DMEM and seeded in the upper chambers, and 500 µL DMEM containing 10% FBS was added to the lower chamber. After incubation at 37°C (Ho8910∶24–26 h; Ho8910-pm:24–26 h; Skov3 24–26 h), the cells were fixed and stained.

### Western blot analysis

The treated cells were lysed with radioimmunoprecipitation assay (RIPA) buffer (50 mM Tris-HCl pH 7.4, 150 mM NaCl, 1% NP-40, 0.5% deoxycholic acid, sodium, 0.1% SDS). Cell lysates were separated by 7.5–12.5% SDS-PAGE, transferred to a nitrocellulose membrane (Bio-Rad,USA), and blocked with PBS containing Tween-20 and 5% non-fat milk for 1 h. Proteins of interest were incubated with corresponding primary antibodies overnight at 4°C. They were then washed three times with washing buffer (0.1% Tween-20 in Tris-buffered saline) and incubated with the appropriate secondary antibody at room temperature for 1 h. The antibody complex was detected using enhanced chemiluminescence Kit (Pierce, Rockford, 1 L. USA). The following primary antibodies SOX2, FAK, phospho-FAK(Y397), Src, phospho-Src(Y416), p130cas, phospho-p130cas, Erk1/2, phospho-Erk1/2, MMP2 and MMP9, were purchased from Cell Signal Technology(Danvers, MA, USA).

### Statistical Analysis

All results are presented as the mean ± standard error of the mean. Statistical analyses were carried out with Fisher's exact test in Table 1. For survival analysis, Kaplan–Meier survival curves were constructed and differences between them were tested by the log-rank test. Otherwise, differences between groups were analyzed using Student's t-test (two-tailed). *p*<0.05 was considered statistically significant.

The article "SOX2 Enhances the Migration and Invasion of Ovarian Cancer Cells via Src Kinase" was retracted in 2023. Reasons: errors in the images; duplicated images; overlap with earlier publications; original data or images not available.

**Table 1:** Correlations between clinicopathological characteristics and expression of SOX2.

Variables	Cases (N)	score of SOX2 expression				*p*
		−	+	++	+++	
Age(year)						
≤60	38	6	8	17	7	0.786
>60	26	3	4	15	4	
Location						
Primary	64	9	12	32	11	0.044*
Metastases	64	7	8	24	25	
Differrentiation						
G1#	2	0	1	1	0	0.006*
G2	31	6	9	14	2	
G3	31	3	2	17	9	
Serum CA125(ng/ml)						
≤800	36	5	7	18	6	0.998
>800	28	4	5	14	5	

# statistics after incorporating of the G1 into G2. *p* value represents the probability from Fisher's exact test for SOX2 expression status between variable subgroups. *, *p*<0.05.

## Results

### Expression of SOX2 in primary tumors and corresponding metastatic lesions in SOC

Ovarian cancer tissue samples from 64 patients were used in this study, and the expression of SOX2 was analyzed in these tissues by using immunohistochemical (IHC) staining. As shown in Table 1, 21 out of 64 (32.8%) of primary lesion tissues had relatively low expression levels of SOX2 protein, whereas 15 out of 64 (23.4%) of the metastatic tissues showed low expression of SOX2 protein. However, 43 out of 64 (67.2%) of primary lesion tissues had relatively high expression levels of SOX2 protein, whereas 49 out of 64 (76.6%) of metastatic tissues showed high expression levels of SOX2 protein. Notably, the expression levels of SOX2 were higher in metastatic lesions than those in their paired primary tumor tissues (Figure 1A and Figure 1B).

**Figure 1:** Overexpression of SOX2 protein in ovarian cancer is correlated with tumor metastasis and prognosis. (**A**), (**B**)Represent two examples of 64 cases. Among A, the upper left represents a primary cancer tissue;the lower left represents the corresponding metastases (omentum). Right, magnification of tissues in black frame. The arragement of B is similar to A. (**C)**, (**D**) Kaplan-Meier survival curves analysis shows subject with high SOX2 expression level have greater risk for death. Ovarian cancer tissues with SOX2 expression(score≥3) were classified as SOX2 high level. Among C, Patients with SOX2 high level(n = 43) had significantly worse survival than those with SOX2 low level(n = 21) in SOC primary tissue(*p* = 0.0358, log-rank test). Among D, Patients with SOX2 high level(n = 49) had significantly worse survival than those with SOX2 low level(n = 15) in SOC metastatic tissue(*p* = 0.0029, log-rank test).

The article "SOX2 Enhances the Migration and Invasion of Ovarian Cancer Cells via Src Kinase" was retracted in 2023. Reasons: errors in the images; duplicated images; overlap with earlier publications; original data or images not available.

The correlations between SOX2 expression and clinical pathological factors in human SOC were further investigated. Interestingly, we found that SOX2 expression was significantly associated with histological grade. Specifically, the SOX2 expression was relatively high in less differentiated tumors (Table 1). The positive staining of SOX2 increased gradually from G2 to G3 grade, indicating that SOX2 protein was increased during the development of SOC. Otherwise, there was no significant associations between the SOX2 expression and age or serum CA125 levels.

The association of SOX2 expression with OS (overall survival) durations and rates at different months was studied. Patients with high-level SOX2 expression had shorter OS durations than those with low-level SOX2 expression in primary tumor tissue and metastatic tissue, respectively (Figure 1C and 1D). Together, these findings suggested that the expression of SOX2 might predict poor prognosis in human ovarian carcinoma.

### SOX2 increases the migratory and metastatic potentials and decreases adhesion ability of SOC cells

To choose suitable cell lines to study the biological function of SOX2, we first analyzed the protein levels of the SOX2 in six ovarian tumor cell lines. We found that the protein levels of SOX2 were greatly varied in different ovarian cancer cell lines. As shown in Figure 2A and Figure 2B, the expression of SOX2 was relatively increased in Skov3 and the highly metastatic cell line Ho8910-pm compared with its parent ovarian cancer cell line Ho8910. The expression of SOX2 was relatively low in the benign ovarian serous cystadenoma eternalized cell line MCV152 and the immortal human ovarian epithelial cell line Moody.

**Figure 2:** SOX2 expression in different ovarian tumor cell lines. Semi-quantitative RT-PCR analysis of SOX2 in six ovarian tumor cell lines. (B) Western blot analysis of the SOX2 protein expression in corresponding cell lines. GAPDH was used for normalization. (C) Semi-quantitative RT-PCR analysis and Western blot analysis of SOX2 in Ho8910-SOX2,Ho8910-pm-siSOX2,Skov3-siSOX2 cells. GAPDH was used for normalization.

To further investigate the function of SOX2 in SOC cells, the SOX2 gene was overexpressed by lentiviral infection in Ho8910, which was confirmed by real-time PCR and Western blotting (Figure 2C). Subsequently, we determined the effect of SOX2 overexpression on the proliferation of the SOC cells. The results showed that overexpression of the SOX2 gene could promote SOC cell proliferation (Figure 3A and Figure 3B). Furthermore, we examined the effect of SOX2 overexpression on the migratory, invasive and adhesive abilities of the SOC cells using transwell assays and cell-ECM adhesion assays. The results showed that overexpression of SOX2 protein could significantly promote the migration and invasion of SOC cells (Figure 4A), while decreasing the adhesion of SOC cells to Matrigel, fibronectin, type I collagen and laminin(Figure 5A).

The article "SOX2 Enhances the Migration and Invasion of Ovarian Cancer Cells via Src Kinase" was retracted in 2023. Reasons: errors in the images; duplicated images; overlap with earlier publications; original data or images not available.

**Figure 3:** SOX2 positively regulates tumor cell proliferation and clone formation. Stable transfection of SOX2 plasmid promote cell proliferation and clone formation (A) CCK8 assays in HO8910. (B) Clone formation assays in HO8910. Transient transfection of SOX2 siRNA inhibit cell proliferation and clone formation (C) CCK8 assays in HO8910-pm. (D) Clone formation assays in HO8910-pm. (E) CCK8 assays in Skov3. (F) Clone formation assays in Skov3.

**Figure 4:** SOX2 promotes cell migration and invasion in SOC cells. (A) Stable transfection of SOX2 plasmid in HO8910. Top, transwell migration assays; Bottom, transwell invasion assays. (B) Transient transfection of SOX2 siRNA in HO8910-pm. Top, transwell migration assays; Bottom, transwell invasion assays. (C) Transient transfection of SOX2 siRNA in Skov3. Top, transwell migration assays; Bottom, transwell invasion assays.

**Figure 5:** SOX2 decrease adhesion in SOC cells. (A) Decrease adhesion after stable transfection of SOX2 plasmid in HO8910. (B) Increase adhesion after transient transfection of SOX2 siRNA in HO8910-pm. (C) Increase adhesion after transient transfection of SOX2 siRNA in Skov3.

Next we knocked down the expression of the SOX2 gene using transient transfection of siRNAs in two cell lines with relatively high expression of SOX2, Ho8910-pm and Skov3. The interference efficiency was confirmed by real-time PCR and Western blotting (Figure 2C). Subsequently, the effect of knockdown of SOX2 on the proliferation of these cells was determined using CCK-8 assays and clone formation assays. The results showed that disruption of SOX2 protein decreased the proliferation of these SOC cells (Figure 3C–3F). Furthermore, we found that knockdown of SOX2 protein expression inhibited the migratory and invasive abilities of SOC cells by transwell assays (Figure 4B and Figure 4C), while promoting the cell adhesion to Matrigel, fibronectin, type I collagen and laminin (Figure 5B and Figure 5C). Taken together, these results suggested that the SOX2 gene may have an important role in the cell proliferation, migration, invasion and adhesion of SOC cells.

### Overexpression of SOX2 leads to increased phosphorylation of multiple pro-matastatic proteins

We further explored the molecular mechanisms underlying SOX2-mediated cell migration and tumor metastasis. We found that stable overexpression of SOX2 resulted in increased phosphorylation of Src and FAK and their downstream molecules (p130-cas) in Ho8910 cells (Figure 6). Moreover, targeted knockdown of the SOX2 gene led to a reduced phosphorylation of these proteins in Ho8910-pm and Skov3 cells (Figure 6).

The article "SOX2 Enhances the Migration and Invasion of Ovarian Cancer Cells via Src Kinase" was retracted in 2023. Reasons: errors in the images; duplicated images; overlap with earlier publications; original data or images not available.

**Figure 6:** SOX2 regulate phosphorylation level of multiple pro-matastatic proteins. (A)Left, western blot analysis proteins expression after stable transfection of SOX2 plasmid in ho8910. Middle, western blot analysis proteins expression after transient transfection of SOX2 siRNA in HO8910-pm. Right, western blot analysis proteins expression after transient transfection of SOX2 siRNA in Skov3. (B) The arragement of B is similar to A.

### Knockdown of Src promotes cell adhesion and decreases cell migration and invasion

The above results suggested that the activation of the Src kinase may be responsible for the tyrosine phosphorylation of p130-cas in SOC cells. To determine whether the Src kinase activity is required for SOX2-induced phosphorylation of p130-cas, we knocked down the Src gene by siRNA in Ho8910-vector and Ho8910-SOX2 cells. The interference efficiency was confirmed by Western blotting (Figure 7B). We found that knockdown of Src protein expression inhibited the migratory and invasive abilities of Ho8910-SOX2 cells in transwell assays (Figure 7A), while promoting the cell adhesion to matrigel, fibronectin, type I collagen, but not laminin (Figure 7C). Furthermore, we found that the phosphorylation of p130-cas could be attenuated in Ho8910-SOX2 cell by knockdown of the Src gene (Figure 7B). Together, these results indicated that the Src kinase activity is essential for SOX2-mediated adhesion and migration of SOC cells.

**Figure 7:** Transient transfection of Src siRNA decrease cell migration and invasion and increase adhesion in HO8910-SOX2 cells. (A) Transwell migration and invasion assays. (B) Western blot analysis proteins expression (C) Adhesion assay.

## Discussion

SOX2 is a key regulator for maintaining the pluripotency and self-renewal of embryonic stem cells and contributes to the reprogramming of differentiated somatic cells back to a pluripotent stem cell state. More recently, enhanced SOX2 expression has been detected in several malignant tumors suggesting that SOX2 also regulates tumorigenesis [3]–[10]. Numerous studies have shown that high expression of SOX2 is correlated with lymphatic and vascular invasion, poor differentiation, and decreased disease-free survival [3]–[8].

Although the association of SOX2 expression with the poor clinical outcome of ovarian cancer has been reported [11], [12], the functional roles and mechanisms in this tumor were less conducted previously, especially in tumor metastasis and adhesion. In our study, SOX2 overexpression promoted cell proliferation and clone formation. However the result is not fully consistent with previous reports [13], [14]. This may be due to the different ovarian cancer cell lines used. Recently, it has been reported that SOX2 targets fibronectin to promote cell migration and invasion in ovarian cancer [14]. In the present study, we found that the Src kinase may be associated with SOX2-induced changes in ovarian cancer. Increased invasion may be related to the increased phosphorylation of multiple pro-metastatic proteins induced by SOX2 overexpression.

The article "SOX2 Enhances the Migration and Invasion of Ovarian Cancer Cells via Src Kinase" was retracted in 2023. Reasons: errors in the images; duplicated images; overlap with earlier publications; original data or images not available.

Src kinase is a non-receptor tyrosine kinase and is known to play essential roles in various signaling pathways of proliferation, migration, adhesion, and angiogenesis during tumor development and progression [17], [18]. Src kinase is overexpressed or activated in several solid tumors, including breast cancer [19], prostate cancer [20], colon cancer [21], gastric cancer [22] and pancreatic cancer [23]. Moreover, it has been shown that Src was associated with the SOX2 expression and self-renewal of stem-like side-population cells in non-small cell lung cancer [24]. Although metastasis is a multifactorial process, invasion is a critical link for tumor cells to metastasize. In the present study, we found that stable overexpression of SOX2 resulted in obviously increased phosphorylation of Src and increased invasion ability, whereas knockdown of the SOX2 gene led to reduced phosphorylation level of Src and invasion ability in SOC. Subsequently, the invasion ability was also decreased following the knockdown of SOX2 or Src.

p130cas can be phosphorylated by Src or FAK family kinases. It acts as a scaffolding molecule to regulate protein complexes that control cell migration and adhesion, apoptosis, cell cycle, differentiation and even progenitor cell function [25], [26], [27]. In this study we also found that the phosphorylation level of p130cas was regulated by Src kinase in SOC lines.

The control of cell-matrix adhesion also plays an important role in controlling cancer cell migration during metastasis [28]. In the early stage of tumor metastasis, reduced adhesion ability of cancer cells will cause cancer cell shedding and invasion to other sites. In our study, adhesion reduction may be also due to the increased expression of matrix metalloproteinases (MMP2 and MMP9) followed by overexpression of SOX2. Fak promoted the formation of the Src-p130cas-Crk-Dock180 signaling complex, leading to the selective elevation of Ras GTPase and JNK, and resulted in increased MMP2 and MMP9 expression [29]. We found that knockdown of Src gene expression can reduce the expression of MMP2 and MMP9. MMP2 and MMP9 are the important metalloproteinases which degrade the ECM and reduce cell adhesion ability. Another cause of adhesion reduction may be due to the increased phosphorylation level of Src and Erk. One study has showed that Src overexpression can inhibit the protein expression level of the integrin subunit by Erk in colon tumor cells [30]. So we deduced that Src overexpression can change the expression or function of the integrin subunit in ovarian cancer cells. This also explains why high expression of FN induced by SOX2 overexpression in ovarian cancer [14], did not lead to adhesion enhancement [31], but a lower adhesion in our study. In our study SOX2 modulated SOC adhesion to matrigel, fibronectin, type I collagen, not including laminin. Specific mechanisms need be further studied.

The article "SOX2 Enhances the Migration and Invasion of Ovarian Cancer Cells via Src Kinase" was retracted in 2023. Reasons: errors in the images; duplicated images; overlap with earlier publications; original data or images not available.

In the present study, we found that one of the mechanisms by which SOX2 promoted SOC cell migration and tumor metastasis is through the phosphorylation and activation of p130cas and high expression of MMP2 and MMP9. It has been well documented that Src family kinases are the major kinases that promote the tyrosine phosphorylation of p130cas and increase expression of MMP2 and MMP9 [26], [32], [33]. Together, we found that SOX2-induced phosphorylation and activation is partly dependent on the activation of Src kinase.

In conclusion, our findings suggested that the SOX2 plays a pivotal role in SOC cell migration and tumor metastasis, and the Src kinase signaling cascade may be a key component of the SOX2 pro-metastatic signaling network in SOC cells.
